The article "Application of Grey-Based SWARA and COPRAS Techniques in Disease Mortality Risk Assessment" was published in 2021. Journal: J Healthc Eng.

# Application of Grey-Based SWARA and COPRAS Techniques in Disease Mortality Risk Assessment

**DOI:** 10.1155/2021/7302157

**Published:** 2021-11-30

**Authors:** Shazia Rehman, Nadia Rehman, Mehvish Naz, Ayesha Mumtaz, Zhang Jianglin

**Affiliations:** ^1^Department of Dermatology, Shenzhen People's Hospital, The Second Clinical Medical College, Jinan University, The First Affiliated Hospital, Southern University of Science and Technology, Shenzhen 518020, Guangdong, China; ^2^Candidate Branch of National Clinical Research Center for Skin Diseases, Shenzhen, China; ^3^Department of Biomedical Sciences, Pak-Austria Fachhochschule, Institute of Applied Sciences and Technology, Haripur, Pakistan; ^4^Department of Mathematics, COMSATS University Islamabad, Wah Campus, Islamabad, Pakistan; ^5^College of Public Administration, Zhejiang University, Hangzhou, China

## Abstract

The health industry is amongst the most affected systems in terms of multiobjective decision-making, rendering the final solution, vulnerable to errors; however, multicriteria decision analysis (MDCA) emerges as a supportive tool for the process of decision-making. Therefore, the present study seeks to offer an MCDA framework for assessing and identifying the potential influence of socioeconomic risk factors on noncommunicable disease mortality. We adopted a subjective approach of grey-based Step-wise Weight Assessment Ratio Analysis (SWARA) and COmplex PRoportional Assessment (COPRAS) approach to calculate weights of parameters and criteria, respectively, and then rank them based on their degree of significance. The findings reveal that CRD mortality is potentially affected by the selected socioeconomic risk variables followed by IHD and cancer. Implementing MCDA techniques in the present study will assist the public health practitioners and policymakers in drawing decisions on the best strategy to reduce CRD mortality, which contributes significantly to raising overall mortality.

## 1. Introduction

A population's health status can be grossly evaluated by measuring death rates. However, a focus on morbidity brings little insight into the burden of diseases that affect population health but do not lead to death. Quantifying health outcomes through both longevity and morbidity offers a more comprehensive view of health outcomes. When the global population rises, life expectancy is increasing, and living standards are improved, and causes of death are changing around the world. Such causes of death vary significantly across the world, depending on country and income levels. A silent pandemic of chronic diseases is progressively engulfing the world's population, spreading across the globe. A distinct continuum of human afflictions gradually replaces infectious and bacterial infections as the world's leading cause of morbidity and mortality, presenting one of the greatest challenges to public health of all time [1, 2].

Noncommunicable diseases (NCDs) remain the major public health concern across the world, causing significant death and morbidity. NCDs are the major causes of mortality and disability around the world. It is estimated that by 2030, these diseases would be responsible for seven out of every ten fatalities in developing nations, as well as in developed nations [3, 4]. Rapid urbanization and substantial population transfers from rural to urban regions are important features of the developmental transition. Even rural residents are gradually adjusting to metropolitan lifestyles. Obesity, cancer, stress, obesity, atherosclerosis, and other NCDs are all caused by a changing lifestyle pattern [5, 6]. Given the projected burden of NCDs and our current health infrastructure, we should reinforce the need of prioritizing NCD prevention and control. Our approaches should be geared toward monitoring the prevalence of NCDs as well as their risk factors. Some NCDs have common risk factors that should be treated with the least cost however the maximum output. The strategy's three main components are monitoring health education and primary prevention. Our social and economic possibilities, such as good public schools, secure employment, and strong social interactions, are crucial for a healthier lifestyle. Employment (work), for example, provides income that influences decisions regarding housing, schooling, child care, food, and healthcare, among other things [7–9]. Unemployment, on the other hand, hinders these alternatives as well as the capacity to amass assets and income that may assist in times of economic difficulty.

The challenge of multiple objectives is constantly present in organizational challenges, raising the complexity towards solutions [10]. In this context, it is important to identify approaches that contain the largest number of factors that guide and impact decisions in the decision-making process to minimize error. However, most of the time, this method is difficult to carry out since, in many circumstances, the decision-making criteria are contradictory, raising the ambiguity in the final response. Decision support techniques, for instance, multicriteria decision analysis (MCDA) methodologies, have evolved to enhance the reliability and legitimacy of the proposed solution [11]. These techniques are designed to aid in decision-making by reducing the responsibility of the ultimate decision-maker and ensuring a solution in compliance with the criteria in issue [12, 13]. In the healthcare domain, these strategies are considerably more complicated as they incorporate not only economic or technical concerns but also the human aspect, which creates a conflict of interest and impedes final decisions [14]. As a result, much research utilizing MCDA is conducted to enhance health systems as a whole [15, 16].

MCDA facilitates a framework for disintegrating a complicated decision into simpler, more manageable components, as well as establishing and comprehending the relationships between them. Measuring each component separately and then combining them to obtain a solution is optional. MCDA also facilitates the complex decision of identifying different priorities and opinions while establishing transparency of the relationship between assessments and optimal solutions [11]. Some investigations have focused on examining a single application sector, like health technology evaluation [17]. Others use a more compassionate approach, reviewing research aimed at determining patient desire [18]. Some go even farther, aiming to fully understand and evaluate the MCDA in health [19]. Given the abundance of research using MCDA in the healthcare setting, the purpose of this study is to offer an MCDA framework that analyzes and identifies the kind of disease mortality that is potentially impacted by socioeconomic variables. We considered ten criteria (socioeconomic factors) to examine the influence on 4 parameters (mortality). Grey Step-wise Weight Assessment Ratio Analysis (SWARA-G) is adopted to compute the weights of the four parameters. Then, we employed Grey COmplex PRoportional Assessment (COPRAS-G) to determine the weight of each selected criterion against each parameter and rank them based on their utility degree. The current study is the first to propose an MCDA approach for identifying the type of disease mortality that may be impacted by socioeconomic variables. Further, the suggested model provides a valuable tool and additional practical knowledge for public health policy and decision-makers in drawing rational decisions to reduce mortality from NCDs affected by socioeconomic factors. For a better understanding, the research theme is presented in Figure 1.

## 2. Research Methodology

### 2.1. Dataset

Following a thorough assessment of prior research on NCD mortality and related risk variables, we considered four parameters in terms of mortality associated with stroke, ischemic heart disease (IHD), chronic respiratory disease (CRD), and cancer. We selected ten socioeconomic risk factors: educational level, gross domestic production (GDP) per capita, energy access, income inequality, economic inequality, inflation, poverty, unemployment, life expectancy, and fertility rate. The steps involved in the computation of grey-based SWARA and COPRAS techniques are calculated using MS Excel.

### 2.2. Grey Numbers

A grey number represents an interim with unspecified information but a well-defined range of possibilities which is depicted by a sign ⊗. In the GST, there are multiple forms of grey numbers; however, the present study introduces the following three forms:

 
*Description 1.* If ⊗*E* is a grey number whose lower limit can only be evaluated, it is termed a grey number with a lower limit only and is expressed as $⊗E=\left[\underline{E},\;\infty \right)$
 
*Description 2*. If ⊗*E* is a grey number whose upper limit can only be evaluated, it is termed a grey number with an upper limit only and is expressed as $⊗E=\left(\infty ,\;\bar{E}\right]$
 
*Description 3*. If ⊗*E* is a grey number whose lower and upper limit can only be evaluated, it is termed an interval grey number and is expressed as $⊗E=\;\left[\underline{E}\;,\;\bar{E}\;\right]$

Let $⊗E=\;\left[\underline{E}\;,\;\bar{E}\;\right]\text{ and}⊗H=\;\left[\underline{H}\;,\;\bar{H}\;\right]$ be two grey numbers, then arithmetic operations ought to be composed in the manner as follows:

(1) $$\begin{array}{c} ⊗E+⊗H=\;\left[\underline{E}+\underline{H},\;\underline{E}-\bar{H}\right],\\ ⊗E-⊗H=\;⊗E+\;\left(-\;⊗H\right)=\;\left[\underline{E}-\bar{H},\;\bar{E}-\bar{H}\right],\\ ⊗E\;\times \;⊗H=\;\left[Min\;\left\{\underline{EH}\;\bar{E}\;\bar{H}\;\bar{E}\;\underline{HE}\;\bar{H}\right\}\;Max\;\left\{\underline{EH}\bar{E}\;\bar{H}\;\bar{E}\;\underline{HE}\;\bar{H}\right\}\right],\\ \frac{⊗E}{⊗H}=\;⊗E\;\times \;⊗H^{-1}=\;\left[\text{Min }\left\{\;\frac{\underline{E}}{\underline{H}}\frac{\underline{E}}{\bar{H}}\frac{\bar{E}}{\underline{H}}\frac{\bar{E}}{\bar{H}}\right\}\right]\text{ Max }\left\{\frac{\underline{E}}{\underline{H}}\frac{\underline{E}}{\bar{H}}\frac{\bar{E}}{\underline{H}}\frac{\bar{E}}{\bar{H}}\right\}. \end{array}$$

The length of the grey number $⊗E=\;\left[\underline{E}\;,\;\bar{E}\right]$ is introduced by the following equation:

(2) $$\begin{array}{c} R\left(⊗E\right)=\bar{E}-\underline{E}. \end{array}$$

If there are two grey numbers $⊗E=\;\left[\underline{E}\;,\;\bar{E}\;\right]\text{ and }⊗H=\;\left[\underline{H}\;,\;\bar{H}\;\right]$, the degree of grey synthetic assessment between these two numbers can be estimated utilizing the following expression:

(3) $$\begin{array}{c} P\left\{⊗E\;\leq \;⊗H\right\}=\frac{Max\;\left\{0,\;R^{*}-Max\;\left(0,\;\bar{E}\;,\;\underline{H}\right)\right\}}{R^{*}}\;,\;where\;R^{*}=R\left(⊗E\right)+R\left(⊗H\right). \end{array}$$

### 2.3. SWARA-G Method

SWARA is an MCDA technique for determining criteria and subcriterion weights. Keršuliene et al. [20] designed this technique. SWARA is commonly used to address complex MCDA issues in a variety of research fields. In this technique, the most significant criterion is stated first, and the least important one is mentioned last. Respondents (experts) play a significant role in setting parameter weights. This approach enables professionals to determine the significance ratio of parameters throughout the weighting procedure. It is effective in gathering and coordinating expert data [21]. Experts also play a significant role in evaluating the estimated weights. Based on their tacit knowledge and experience, each expert determines the significance of each criterion. The weight of each criterion is then computed based on the average value of group evaluations acquired from experts. In this work, the SWARA technique is utilized to determine parameter weights using grey numbers. The scale of grey numbers with linguistic variables to weight and rank the criteria and alternatives is presented in Table 1.

### 2.4. COPRAS-G Method

To estimate and rank the criteria, Zavadskas et al. [22] proposed the COPRAS-G method. We employ COPRAS-G to rank the criteria in the current study. According to Nguyen et al. [23], this approach evaluates and offers a ranking sequence of criteria based on their importance and degree of utility. The stages involved in this method's computations are as follows:

*Step I.* Determine the evaluation parameter, and the selected parameter should significantly describe the alternatives.
*Step II.* Construct the initial grey decision matrix:
  (4) $$\begin{array}{c} ⊗Y=\left[\begin{array}{ccc} y_{11} & \cdots & ⊗y_{1k}\\ \vdots & \ddots & \vdots \\ ⊗y_{l1} & \cdots & ⊗y_{lk} \end{array}\right]=\left[\begin{array}{ccc} \left[b_{11};c_{11}\right] & \cdots & \left[b_{1k};c_{1k}\right]\\ \vdots & \ddots & \vdots \\ \left[b_{l1};c_{l1}\right] & \cdots & \left[b_{lk};\left[c_{lk}\right]\right] \end{array}\right],\;j=1\cdots l;i=1\cdots k, \end{array}$$
where ⊗*y*_*ji*_ is estimated by *b*_*ji*_ (the least value or the lower limit) and *c*_*ji*_ (the highest value or the upper limit).
*Step III*. Normalize the initial grey decision matrix ⊗*Y* using the following expressions:
  (5) $$\begin{array}{c} \bar{b_{ji}}=\frac{2b_{ji}}{\left(\sum_{j=1}^{l}b_{ji}+\sum_{j=1}^{l}c_{ji}\right)},\\ \bar{c_{ji}}=\frac{2c_{ji}}{\left(\sum_{j=1}^{l}b_{ji}+\sum_{j=1}^{l}c_{ji}\right)}, \end{array}$$
for  *j*=1 ⋯ *l* *an*  *d* *i*=1 ⋯ *k*.
Then, the normalized expression would be as follows:
  (6) $$\begin{array}{c} ⊗\hat{Y}=\left[\begin{array}{ccc} ⊗\bar{y_{11}} & \cdots & ⊗y_{1k}\\ \vdots & \ddots & \vdots \\ ⊗\bar{y_{l1}} & \cdots & ⊗y_{lk} \end{array}\right]=\left[\begin{array}{ccc} \left[b_{11};c_{11}\right] & \cdots & \left[b_{1k};c_{1k}\right]\\ \vdots & \ddots & \vdots \\ \left[b_{l1};c_{l1}\right] & \cdots & \left[b_{lk};c_{lk}\right] \end{array}\right],\;j=\bar{1,l};i=\bar{1,k}. \end{array}$$
*Step IV*. Determine the relative weighting of each assessment parameter. The SWARA-G technique is used in this study to determine the weight of each parameter.
*Step V*. Compute the weighted normalized decision matrix. The normalized decision-making matrix is multiplied by weights generated using the SWARA-G technique in this phase as follows:
  (7) $$\begin{array}{c} ⊗{\hat{y}}_{j1}=⊗{\hat{y}}_{j1}.f_{i};{\hat{b}}_{j1}={\hat{b}}_{j1}.f_{i};\;{\hat{c}}_{j1}={\hat{c}}_{j1}.f_{i}. \end{array}$$
Then, the weighted normalized grey decision matrix is shown as follows:
  (8) $$\begin{array}{c} ⊗\hat{Y}=\left[\begin{array}{ccc} ⊗{\hat{y}}_{11} & \cdots & ⊗{\hat{y}}_{1k}\\ \vdots & \ddots & \vdots \\ ⊗{\hat{y}}_{l1} & \cdots & ⊗{\hat{y}}_{lk} \end{array}\right]=\left[\begin{array}{ccc} \left[{\hat{b}}_{11};c_{11}\right] & \cdots & \left[{\hat{b}}_{1k};{\hat{c}}_{1k}\right]\\ \vdots & \ddots & \vdots \\ \left[{\hat{b}}_{l1};c_{l1}\right] & \cdots & \left[{\hat{b}}_{lk};\left[{\hat{c}}_{lk}\right]\right] \end{array}\right]. \end{array}$$
*Step VI*. Determine the relative significance of each criterion by summing the weighted normalized grey decision matrix as beneficial (*P*_*j*_) and nonbeneficial (*R*_*j*_) attributes individually.
Beneficial attribute $P_{j}=1/2\sum_{j=1}^{l}\left({\hat{b}}_{j1}+{\hat{c}}_{j1}\right)$.
Nonbeneficial attribute $R_{j}=1/2\sum_{j=k+1}^{l}\left({\hat{b}}_{j1}+{\hat{c}}_{j1}\right),\;j=\bar{k,l}$.
*Step VII*. After determining the minimum value from the nonbeneficial (*R*_*i*_) criteria, the relative significance (*S*_*j*_) of each criterion is calculated in such a way that the poorest alternative has the lowest weight priority:
  (9) $$\begin{array}{c} S_{j}=P_{j}+\frac{\sum_{j=1}^{l}R_{j}}{R_{j}\sum_{j=1}^{l}1/R_{j}}. \end{array}$$
*Step VIII*. Determine the maximum weight of the criteria (*S*_*j*_) and then calculate the degree of utility for each criterion by contrasting it to the worst criterion. The degree of utility has a value ranging from 0% (worst) to 100% (best):
  (10) $$\begin{array}{c} D_{j}=\frac{S_{j}}{S_{max}}\times 100\%. \end{array}$$

## 3. Results

In the present analysis, the proposed SWARA-G method is used to weigh four parameters. The weighting steps involved in the computations of the SWARA-G method were described in detail in reference [20]. To calculate the weights, 10 criteria in 4 parameters (stroke, IHD, CRD, and Cancer) are considered. Based on expert judgments, we assigned linguistic variables to selected parameters as presented in Table 1. After assigning the linguistic variables, we converted them into grey numbers and then aggregated them. Based on that we moved to the next step of estimating the coefficient (*C*_*i*_) and then recalculated the weight (*W*_*i*_) for each parameter. The final weights (*F*_*i*_) were calculated which were the input for the next method of COPRAS-G. After performing the SWARA-G method, the weight assigned to each parameter is provided, as shown in Table 2.

### 3.1. COPRAS-G Analysis

The COPRAS-G method provides a ranking procedure against four parameters. The grey weights for each parameter found via the SWARA-G method are the inputs for COPRAS-G. The aggregated initial grey decision matrix, normalized grey decision matrix, and weighted normalized grey decision matrix are expressed in Table 3–5. Educational level, GDP per capita, access to energy, unemployment, life expectancy, and fertility rate are considered as beneficial criteria, whereas income inequality, economic inequality, inflation, and poverty are considered as nonbeneficial criteria for assessing disease burden of stroke, IHD, CRD, and cancer mortality.

Following COPRAS-G, the degree of utility of each parameter (*U*_*i*_) is estimated.  Table 6 presents the ranking order of four parameters based on ten criteria. As shown in Table 6, parameter 3 (CRD) with the utility degree of 57.19% is the worst scenario based on the selected criteria followed by parameter 2 (IHD), parameter 4 (cancer), and parameter 1 (stroke) with the utility degree of 66.32%, 74.18, and 100%, respectively, for mitigating the disease burden due to CRD, IHD, cancer, and stroke. The ranking sequence based on the grey-based COPRAS technique in the schematic diagram is presented in Figure 2.

## 4. Discussion and Conclusions

NCDs have accounted for a significant increase in seven of the world's leading causes of mortality during the last two decades. Social and economic variables can have a huge effect on how healthy we are and how long we survive. These variables influence our capacity to make healthy decisions, afford medical treatment and housing, and deal with stress, among other things [25]. The current analysis evaluates prospective disease mortality from stroke, IHD, CRD, and cancer to social and economic variables using a grey-based MCDA technique. We proposed a technique that comprehensively analyzes the impact of these variables on health outcomes in terms of mortality from various NCDs. Importantly, this study employs a multicriteria decision-making technique to identify which disease mortality is more impacted by the specified risk variables. Our findings show that CRD mortality is most likely to be influenced by the chosen socioeconomic variables, followed by IHD and cancer. Respiratory illnesses are the major cause of mortality and disability worldwide. Chronic obstructive pulmonary disease (COPD) affects around 65 million people globally and kills 3 million people annually, ranking it the third-largest cause of mortality. CRDs are already prevalent in developed nations and are expanding rapidly. Given the global population aging and economic pressures of poor diets and smoking, the rapid expansion of westernized in low- and middle-income nations adds to the rising prevalence of CRDs in these economies. In addition to psychological issues, there is a direct link between poorer health and low income, which adds to food insecurity, the purchase of cheaper and harmful dietary goods, and the cost of expensive therapies. People with modest wages believe they have a lesser social position, which hinders them from engaging in social activities.

There is a rising trend to examine societal and economic structures as significant variables influence CRDs apart from human behavior/lifestyle. Krieger's ecosocial disease distribution hypothesis emphasizes how variety in historical, sociological, and ecological circumstances greatly contributes to differences in the health outcomes of distinct social groups [26, 27]. For example, the current coronavirus COVID-19 epidemic highlights the negative consequences of long-standing economic and health disparities. As per Krieger's study, the greater proportion of COVID-19 deaths in African Americans than whites in the United States is due to a combination of factors such as living in crowded areas, taking public transport services to work, working in service jobs that require direct contact with each other, and a lack of protective equipment at worksites. Furthermore, among the African American community, a lack of healthcare access and medical insurance, as well as pre-existing health problems, may raise the risk of COVID-19 [28].

CRD preventive measures might entail both modest and large-scale human collaboration. The significance of avoiding CRDs stems from their direct influence on the declining rate of national income. Large-scale productivity loss is the result of the incapacity to work and persistent absence risks to the national economy. The CRD prevention strategy is based on risk factor management, which addresses individuals, societies, countries, and the global level through activities such as allocation of resources, multisectoral collaboration, knowledge, and management of information and innovations. The most crucial component of the preventive approach is lifestyle management at the individual level, with an emphasis on behavior, such as innovations, that can assist society in raising awareness of risk factor management, making health policy decisions at the national level, and developing a global health strategy. The significance of leadership in the change management process is emphasized, and new methods to CRD prevention are required [29].

The need for tools that aid in decision-making occurs in a variety of healthcare settings, and these tools are employed to varying degrees in different settings [30, 31]. In this study, we focus on the possibilities of using a specific decision-making assistance technique in disease-related risk variables. Since the evaluation of mortality and morbidity associated risk variables is an innately complex system that cannot be represented using a single metric only, multidimensional analysis and, as a result, multidimensional (MCDA) approaches are highly suggested for this risk assessment [32]. As a result, the goal of our study was to investigate the feasibility of employing the grey-based COPRAS approach to assess and identify possible disease mortality among the selected risk variables. Although the COPRAS technique is arguably the most known and best-detailed ranking method in the literature, the inclusion of grey numbers has extended its application area. The technique presented in this paper is quite simple. Any spreadsheet may be used to execute mathematical operations, which is very important for small sample sizes. The COPRAS-G technique may be successfully utilized in the biomedical domain to analyze, compare, and identify the possible disease burden of mortality and to prioritize them according to their worst scenarios, as shown in the studies and analyses presented here. Utilizing the MCDA techniques in the present study will assist the public health practitioners and policymakers in drawing decisions on the best way to minimize CRD mortality that plays a significant role in raising overall mortality. More importantly, this investigation facilitates researchers with an MCDA roadmap to help them enhance the quality of their studies and their understanding of how to use MCDA techniques to evaluate and prioritize the influencing disease burden of mortality in healthcare research.

Categorically speaking, MCDA is an organized, transparent, coherent, and legitimate way for assisting healthcare decision-making because it facilitates a comprehensive framework to disintegrate a complex structure into a transparent and pragmatic phase that encompasses the relative importance of various perspectives. Real-life examples of appropriate MCDA application in healthcare decision-making in all perspectives to improve the quality of healthcare indicate that MCDA may be employed to support comprehensive assessments. MCDA could be adopted at the macro and micro settings or the hospital and healthcare-provider levels. It is worth noting that the successful application of MCDA is an iterative procedure. It is advised that MCDA be piloted before being widely implemented. MCDA approaches should be extensively considered as a tool to aid healthcare decision-making in order to promote openness, fairness, and teamwork to reach an optimal solution.

## Figures and Tables

**Figure 1:** The study theme.

**Figure 2:** COPRAS-G-based ranking order.

**Table 1:** Linguistic variables and corresponding grey numbers.

Linguistic variables	Grey numbers for rating criteria	Grey number for rating alternatives
Insignificant	[0.0, 0.1]	[0.0, 1.0]
Low	[0.1, 0.3]	[1.0, 3.0]
Medium-low	[0.3, 0.4]	[3.0, 4.0]
Medium	[0.4, 0.5]	[4.0, 5.0]
Medium significant	[0.5, 0.6]	[5.0, 6.0]
Significant	[0.6, 0.9]	[6.0, 9.0]
Very significant	[0.9, 1.0]	[9.0, 10.0]

**Table 2:** Weighting the criteria using the SWARA-G method.

Parameter	Comparative importance of average value *S*_*i*_	Coefficient *C*_*i*_ = *S*_*i*_ + 1	Recalculated weight *W*_*i*_ = *W*_*i*_ − 1/*C*_*i*_	Final weight *F*_*i*_=*W*_*i*_/^∑^*W*_*i*_
Stroke		[1, 1]	[1.00, 1.00]	[0.506, 0.531]
IHD	[0.9, 1.0]	[1.9, 2.0]	[0.526, 0.500]	[0.266, 0.267]
CRD	[0.9, 1.0]	[1.9, 2.0]	[0.277, 0.250]	[0.140, 0.133]
Cancer	[0.6, 0.9]	[1.6, 1.9]	[0.173, 0.132]	[0.088, 0.070]

**Table 3:** The aggregated initial grey decision matrix.

	Educational level	GDP per capita	Access to energy	Income inequality	Economic inequality
Stroke	[7.00, 8.50]	[5.65, 7.50]	[5.90, 7.05]	[4.55, 6.65]	[6.40, 8.60]
IHD	[6.45, 8.25]	[4.75, 6.35]	[6.30, 7.75]	[5.65, 6.85]	[4.45, 7.70]
CRD	[4.55, 5.75]	[5.10, 7.30]	[4.45, 6.55]	[6.55, 8.45]	[4.75, 7.25]
Cancer	[5.75, 7.85]	[4.20, 6.35]	[6.30, 8.25]	[6.20, 8.35]	[5.35, 7.65]

	Inflation	Poverty	Unemployment	Life expectancy	Fertility rate
Stroke	[5.05, 7.85]	[7.00, 8.50]	[5.65, 7.50]	[6.50, 7.55]	[4.25, 6.25]
IHD	[4.30, 6.20]	[4.20, 8.25]	[4.25, 7.30]	[5.25, 7.35]	[4.35, 7.85]
CRD	[5.50, 7.75]	[5.40, 8.45]	[6.55, 8.30]	[4.40, 7.55]	[5.60, 8.75]
Cancer	[4.40, 7.25]	[5.55, 6.80]	[5.20, 8.35]	[6.35, 8.30]	[5.10, 8.65]

**Table 4:** The normalized grey decision matrix.

	Educational level	GDP per capita	Access to energy	Income inequality	Economic inequality
Stroke	[0.259, 0.314]	[0.239, 0.318]	[0.225, 0.268]	[0.171, 0.250]	[0.245, 0.330]
IHD	[0.238, 0.305]	[0.201, 0.269]	[0.240, 0.295]	[0.212, 0.257]	[0.171, 0.295]
CRD	[0.168, 0.213]	[0.216, 0.309]	[0.169, 0.249]	[0.246, 0.317]	[0.182, 0.278]
Cancer	[0.213, 0.290]	[0.178. 0.269]	[0.240, 0.314]	[0.233, 0.314]	[0.205, 0.293]

	Inflation	Poverty	Unemployment	Life expectancy	Fertility rate
Stroke	[0.209, 0.325]	[0.259, 0.314]	[0.213, 0.282]	[0.244, 0.284]	[0.167, 0.123]
IHD	[0.178, 0.257]	[0.155, 0.305]	[0.160, 0.275]	[0.197, 0.276]	[0.171, 0.309]
CRD	[0.228, 0.321]	[0.199, 0.312]	[0.247, 0.313]	[0.165, 0.284]	[0.220, 0.345]
Cancer	[0.182, 0.300]	[0.205, 0.251]	[0.252, 0.315]	[0.238, 0.312]	[0.201, 0.341]

**Table 5:** The weighted normalized grey decision matrix.

	Educational level	GDP per capita	Access to energy	Income inequality	Economic inequality
Stroke	[0.131, 0.167]	[0.121, 0.169]	[0.114, 0.142]	[0.087, 0.133]	[0.124, 0.175]
IHD	[0.063, 0.081]	[0.053, 0.072]	[0.064, 0.079]	[0.056, 0.069]	[0.045, 0.079]
CRD	[0.024, 0.028]	[0.030, 0.041]	[0.024, 0.033]	[0.034, 0.042]	[0.025, 0.037]
Cancer	[0.019, 0.020]	[0.016, 0.019]	[0.021, 0.022]	[0.021, 0.022]	[0.018, 0.021]

	Inflation	Poverty	Unemployment	Life expectancy	Fertility rate
Stroke	[0.106, 0.173]	[0.131, 0.167]	[0.108, 0.150]	[0.123, 0.144]	[0.086, 0.065]
IHD	[0.047, 0.069]	[0.041, 0.081]	[0.043, 0.073]	[0.052, 0.074]	[0.045, 0.083]
CRD	[0.032, 0.043]	[0.028, 0.041]	[0.035, 0.042]	[0.023, 0.038]	[0.031, 0.046]
Cancer	[0.016, 0.021]	[0.018, 0.019]	[0.022, 0.024]	[0.021, 0.026]	[0.018, 0.001]

**Table 6:** The utility degree and corresponding ranking order.

Parameters	*P*_j_	*R*_j_	*Q*_j_	Utility degree (*S*_j_)	Ranking
Stroke	0.760	0.548	0.8314	100	4^th^
IHD	0.391	0.244	0.5514	66.32	2^nd^
CRD	0.198	0.141	0.4755	57.19	1^st^
Cancer	0.115	0.078	0.6167	74.18	3^rd^

## Data Availability

The data used and/or analyzed during the current study is already available from the literature.
